# Influencing Factors and Coping Strategies of Hospitalization in Children with Leukemia Complicated with Pneumonia

**DOI:** 10.1155/2022/4648784

**Published:** 2022-07-15

**Authors:** Rongmei Xiang, Jiang Yi

**Affiliations:** Pediatrics, Hanchuan People's Hospital, Hanchuan, Hubei 431600, China

## Abstract

**Objective:**

To investigate the influencing factors of pneumonia when pediatric leukemia patients are hospitalized and propose coping strategies.

**Methods:**

A retrospective study and analysis of the inpatient medical records of 183 children with leukemia in our hospital from August 2017 to August 2020. A total of 93 cases were in the case group of children with pneumonia, and the rest were 90 cases in the control group. Case data from two groups of children were compared, and the monofactor analysis of pneumonia occurred. The *P* < 0.05 was selected for its multivariate logistic regression analysis, and its coping strategy was proposed.

**Results:**

After multivariate logistic retrospective analysis, it was found that the main influencing factors were neutrophils, white blood cells, vitamin D, and cellular immunity (*P* < 0.05). A review of the two sets of pathological data found that high doses of cytarabine reduced the incidence of pneumonia in children with leukemia (*P* < 0.05).

**Conclusion:**

A timely understanding of the influencing factors of pediatric diabetes mellitus and pneumonia and the early application of cytarabine can reduce the incidence of pneumonia during the child's hospitalization.

## 1. Introduction

Pediatric leukemia is a common malignancy in childhood, resulting from hematopoietic stem cell mutation due to various pathogenic factors, and it seriously threatens the health of children [1]. The main manifestations are fever, bleeding, and lymphadenopathy. The main causes of the disease are viral factors, ionizing radiation, chemical factors, etc., and the 5-year survival rate of children after the illness has reached 70.8% [2]. In China, the mortality rate of pediatric leukemia ranks first, and the incidence rate is also increasing year by year [3]. Leukemia is a malignant clonal hematopoietic system disease; the main characteristics are characterized by the long course, high difficulty in the cure, rapid onset of disease, and high medical costs, which not only adversely affect the physical health of the child but also increase his family and socioeconomic burden. In addition, the children are younger, and they are also prone to adverse psychological states during treatment [4]. Its main treatment methods are chemotherapy, targeted therapy, antitumor drugs, and hematopoietic stem cell transplantation. Chemotherapy is the main way to treat leukemia. Through chemotherapy, abnormal white blood cells are cleared to rebuild normal bone marrow cells [5], which plays a key role in improving the survival rate or cure of children. However, long-term chemotherapy can lead to bone marrow suppression, agranulocytosis, and decreased body immunity. At the same time, due to the immature development of the child's autoimmune and respiratory tract reasons, the spread of pathogens through the air into the child will lead to an increase in the rate of infection, which is one of the critical causes of treatment failure or death [6]. Clinically, concomitant pneumonia is more common because it is difficult to judge in the early stage of concomitant pneumonia, the course of the disease is long, and the prognosis is poor [7]. Therefore, early prevention and effective control are the key points to improve the survival rate and cure rate of children. This study investigated the influencing factors during hospitalization of patients with pediatric leukemia complicated with pneumonia and proposed coping strategies to provide an objective basis for prevention and treatment.

## 2. Information and Methods

### 2.1. Research Subjects

A retrospective study was conducted on the inpatient medical records of 183 children with leukemia admitted to our hospital from August 2017 to August 2020. A total of 93 cases were in the case group of children with pneumonia, and the remaining 90 cases were in the control group. The case group had 51 males and 42 females, aged 1-4 years, with an average age of 6.4 ± 1.7 years. There were 48 males and 42 females in the control group, with an age of 1 to 4 years and a mean age of 7.1 ± 1.3 years. None of the patients dropped out of the study halfway through.

Inclusion criteria are as follows: (1) meet the diagnostic criteria for leukemia [8], (2) meet the WS382 pneumonia diagnostic criteria [9], (3) age 1 to 14 years old, (4) complete medical records and treatment in our hospital, and (5) informed consent; this study was approved by the ethics society. Exclusion criteria are as follows: (1) children with distant tumor metastasis, recurrence, and multiple organ failure; (2) children with expected survival time ≤ 1 month; (3) combined with other immune-related diseases and genetic metabolic diseases; (4) patients with incomplete clinical data; and (5) patients who dropped out of the study midway.

### 2.2. Methods

Refer to the relevant literature and the opinions and suggestions of the chief physician of pediatrics, hematology, and infectious diseases to include factors that may affect the occurrence of pneumonia in children with leukemia, including personal history, disease and treatment history, routine blood tests, and immune function tests. Personal history includes basic information (sex, age, height, and weight) and monthly income. History of illness and treatment includes leukemia typing, number of chemotherapy cases, drug use status, and bone marrow/lumbar puncture. Past history, that is, past infection and the number of infections, was made into a questionnaire. The content validity was evaluated by one chief physician of pediatrics, hematology, and infectious diseases, and the content validity index (CVI) = 0.94. The main family caregivers of the patients responded and recorded and surveyed their responses to determine their reliability.

### 2.3. Statistical Analysis

SPSS 23.0 was used to analyze and process the data, and the data conforming to the normal distribution were expressed as mean ± standard deviation ($\bar{x}\pm s$). The *t*-test calculates the classification, the nonnormal distribution data is expressed as a percentage (%), and the *χ*^2^ test is performed. The factors with statistical significance (*P* < 0.05) were selected, and a multivariate logistic regression analysis was performed to screen out the main influencing factors. The test level was taken as *a* = 0.05. *P* < 0.05 indicated that the difference was statistically significant.

## 3. Results

### 3.1. Monofactor Analysis of Clinical Data

The analysis of clinical data of the two groups of patients showed that the use of high-dose cytarabine drugs, leukocytes, neutrophils, platelets, hemoglobin, vitamin D, CD3^+^ CD4^+^, and CD3^+^ CD8^+^ and other 8 factors between the case group and the control group had significant statistical differences (*P* < 0.05). These factors may be associated with pneumonia in children with leukemia. No significant differences exist in the remaining personal history, disease and treatment history, and immune function testing (*P* > 0.05). See Table 1.

### 3.2. Multivariate Logistic Regression Analysis

The single factor with statistical significance was screened through monofactor analysis, the independent variable was assigned, and a multivariate logistic regression analysis was performed. The methods are visible in Table 2.

After the assignment, the second multivariate logistic regression analysis was performed for the monofactor analysis, and one protective factor was screened out. The OR value of the use of high-dose cytarabine is 0.374 (*P* < 0.05). Four risk factors were leukocytes, neutrophils, vitamin D, and cellular immunity (CD3^+^ CD4^+^, CD3^+^ CD8^+^); OR values were 4.775, 4.384, 3.629, 3.504, and 3.575, respectively (*P* < 0.05). See Table 3.

## 4. Discussion

Pediatric leukemia is a more common form of the chronic hematologic disorder that is more common than pneumonia during treatment. As children receive long-term chemotherapy and broad-spectrum antibiotic therapy, more and more children with leukemia have pneumonia. Studies have shown that the incidence of pneumonia is as high as 25% to 50% [10]. The main clinical symptoms are fever, shortness of breath, etc. Most children lack other symptoms and positive signs. Therefore, early detection of risk factors can reduce the incidence of pneumonia.

Most routine blood tests for pediatric leukemia show decreased white blood cells and neutrophils. The main functions of neutrophils are chemotaxis, phagocytosis, and sterilization. In this series, leukocytes complete functions such as adhesion, crossing the vascular endothelium, and exuding from the site of inflammation [11]. The case group's white blood cell and neutrophil counts were significantly lower than those in the control group. Multivariate logistic regression analysis showed that the neutrophil OR value was 4.384 (*P* < 0.05) and the leukocyte OR value was 4.775 (*P* < 0.05), indicating that neutrophils and leukocytes were risk factors for pediatric leukemia with pneumonia. Vitamin D is not only one of the fat-soluble vitamins that can promote the growth and development of the human body and maintain the balance of calcium and phosphorus, but it also has immunomodulatory functions. It can be activated in the lungs to stimulate antibiopeptide expression sequences in neutrophils, macrophages, monocytes, and respiratory epithelial cells. It has a certain degree of antilung infection effect, strengthens macrophages, and improves their bacteriophage capacity [12, 13]. The results of the monofactor analysis of this study showed that the content of vitamin D was significantly different between the two groups, and the multivariate logistic regression analysis showed that the OR value of vitamin D was 3.629. This indicates that vitamin D is an independent risk factor for pediatric leukemia with pneumonia. Lymphocyte surface antigens constitute the main immune system in the body and respond to the body's cellular immunity level through CD3^+^ CD4^+^ and CD3^+^ CD8^+^, which can directly reflect the body's cellular immune function state [14]. The body's cellular immune function will be disrupted in the chemotherapy and hormone therapy process, resulting in a decrease in immunity [15]. In this study, the cellular immune function of both the case group and the control group decreased, and the decline was more obvious in the case group. In the multivariate logistic regression analysis, the CD3^+^ CD4^+^ and CD3^+^ CD8^+^ OR values were 3.504 and 3.575, respectively, which suggests that cellular immunocompromise is an independent risk factor for pediatric leukemia with pneumonia. The proportion of high-dose cytarabine drugs used in the control group was 70.00% during the hospitalization of the children, and the proportion of the case group was 47.31%. A multivariate logistic regression analysis was performed after the assignment of its independent variables. Its OR value was 0.374, indicating that the use of high-dose cytarabine drugs was a protective factor for pediatric leukemia with pneumonia. As one of the drugs for the treatment of leukemia, cytarabine drugs can inhibit cell DNA synthesis, promote interference in cell proliferation, have antiviral effects, and reduce the incidence of pneumonia in children [16, 17].

Therefore, at the beginning of the disease, health education, strengthening health protection, avoiding spicy and irritating foods, doing oral care, bed rest, and preventing skin and mucous membrane damage are very important. During hospitalization, due to the damage caused by long-term chemotherapy to the body's immunity, it is important to keep the ward clean and disinfected, to treat the child separately from the child with pneumonia, to prevent cross-infection during the diagnosis and treatment of medical staff, and to strictly follow the principle of sterile operation [18]. There are also some shortcomings in this study, where the patients in this study are all from the same hospital, which can lead to some bias in the results. At the same time, the sample size of this study is small and not strongly representative, so it still needs to be further verified by large-sample size studies.

In summary, the risk factors for pediatric leukemia with pneumonia during hospitalization include leukocytes, neutrophils, vitamin D, and cellular immunity, and the protective factor is the use of high-dose cytarabine drugs. Therefore, children with leukemia should be treated with pneumonia in the early stage of the disease, understand the influencing factors of pediatric diabetes mellitus and pneumonia, and deal with it correctly. Early application of cytarabine drugs and active implementation of coping strategies reduce the incidence of pneumonia during the child's hospitalization.

## Figures and Tables

**Table 1:** Clinical data analysis results.

Monofactor	Case group (*n* = 93)	Control group (*n* = 90)	*t*/*χ*^*2*^ value	*P* value
Personal history				
Age (years)	6.8 ± 1.7	7.1 ± 1.3	1.337	0.182
Weight (kg)	18.4 ± 2.5	18.6 ± 2.4	0.551	0.581
Gender (male/female)	51/42	48/42	0.042	0.838
Height (m^2^)	1.04 ± 0.53	1.05 ± 0.51	0.130	0.896
Monthly income (yuan)	4539.63 ± 517.94	4544.04 ± 515.32	0.057	0.954
Disease and treatment history				
Acute lymphoblastic leukemia (*n*, %)	88 (94.62)	86 (95.55)	0.085	0.771
Number of cases receiving chemotherapy (*n*, %)	91 (97.84)	87 (96.66)	0.241	0.624
Use of anthracyclines (*n*, %)	53 (56.98)	51 (56.66)	0.002	0.965
Use of high-dose cytarabines (*n*, %)	44 (47.31)	63 (70.00)	9.696	0.002
Use of glucocorticoid drugs (*n*, %)	37 (39.78)	31 (34.44)	2.981	0.084
Bone marrow/lumbar puncture (*n*)	16/12	17/14	0.032	0.859
Blood routine examination				
Leukocytes (×10^9^/L)	2.37 ± 1.48	5.84 ± 5.27	6.106	<0.001
Neutrophils (×10^9^/L)	0.47 ± 0.41	0.91 ± 0.52	6.381	<0.001
Platelets (×10^9^/L)	34.2 ± 28.15	48.4 ± 21.82	3.805	0.002
Hemoglobin (g/dL)	67.1 ± 15.64	75.61 ± 19.11	3.301	0.001
Vitamin D (ng/mg)	13.64 ± 6.41	16.61 ± 8.63	2.648	0.008
Immune function test				
CD3^+^ CD4^+^	20.4 ± 1.64	22.85 ± 7.35	3.088	0.002
CD3^+^ CD8^+^	23.63 ± 9.66	18.6 ± 11.09	3.274	0.001
IgM (g/L)	1.06 ± 0.73	1.32 ± 1.31	1.651	0.097
IgA (g/L)	1.07 ± 0.72	1.43 ± 1.65	1.923	0.056
IgG (g/L)	9.65 ± 3.44	9.46 ± 4.21	0.334	0.738

**Table 2:** Results after argument assignment.

Monofactor	Variable	Value assignment
High-dose cytarabine drugs are used	X1	Yes = 1, no = 0
Leukocytes	X2	5.5 ~ 3.5 × 10^9^/L = 1, 3.5 ~ 1.5 × 10^9^/L = 2, <1.5 × 10^9^/L = 3
Neutrophils	X3	0.5 ~ 1.5 × 10^9^/L = 1, 0.2 ~ 0.5 × 10^9^/L = 2, <0.2 × 10^9^/L = 3
Platelets	X4	100 ~ 80 × 10^9^/L = 1, 80 ~ 50 × 10^9^/L = 2, <50 × 10^9^/L = 3
Hemoglobin	X5	12 ~ 11 = 1, 11 ~ 10 = 2, <10 = 3
Vitamin D	X6	26 ~ 15 = 1, 15 ~ 10 = 2, <10 = 3
CD3^+^ CD4^+^	X7	25 ~ 15 = 1, 15 ~ 10 = 2, <10 = 3
CD3^+^ CD8^+^	X8	30 ~ 20 = 1, 20 ~ 10 = 2, <10 = 3

**Table 3:** Variables do not enter the regression model.

Variable	*β*	*P*	OR	SE	95% CI
X1	-0.981	0.039	0.374	0.487	0.144-0.973
X2	1.564	0.001	4.775	0.675	1.272-17.939
X3	1.778	0.026	4.384	0.682	1.151-16.688
X4	-1.113	0.062	0.328	0.691	0.084-1.272
X5	-1.024	0.237	0.359	0.792	0.076-1.696
X6	1.289	0.009	3.629	0.654	2.201-5.983
X7	1.254	0.037	3.504	0.634	3.259-3.767
X8	1.274	0.048	3.575	0.597	2.093-6.104

## Data Availability

The datasets used and analyzed during the current study are available from the corresponding author upon reasonable request.
